The article "Efficacy of fertilizing method for different potash sources in cotton (Gossypium hirsutum L.) nutrition under arid climatic conditions" was retracted in 2022. Reasons: compromised peer review; a conflict of interest; concerns about the authorship.

# Efficacy of fertilizing method for different potash sources in cotton (*Gossypium hirsutum* L.) nutrition under arid climatic conditions

**DOI:** 10.1371/journal.pone.0228335

**Published:** 2020-01-24

**Authors:** Mubshar Hussain, Ahmad Faizan Tariq, Ahmad Nawaz, Muhammad Nawaz, Abdul Sattar, Sami Ul-Allah, Abdul Wakeel

**Affiliations:** 1 Department of Agronomy, Bahauddin Zakariya University, Multan, Pakistan; 2 Agriculture Discipline, College of Science, Health, Engineering and Education Murdoch University, Murdoch, WA, Australia; 3 College of Agriculture, BZU, Bahadur Sub Campus, Layyah, Pakistan; 4 Institute of Soil and Environmental Sciences, University of Agriculture, Faisalabad, Pakistan; Harran University, TURKEY

## Abstract

Precise choice of potassium (K) source and application method does matter for its cost-effectiveness. This study was aimed to evaluate the best source and method of K fertilizer application to improve cotton productivity and profitability under an arid climate. Three different K sources (KNO_3_, K_2_SO_4_ and KCl) were applied at 100 kg ha^-1^ by four methods, i.e. a) basal application, b) side dressing, c) fertigation and d) foliar application of 2% K_2_SO_4_. The highest productivity and profitability were recorded with K_2_SO_4_ applied as foliar application. Total boll weight per plant was similar in foliar applied K_2_SO_4_ and basal application of KNO_3_. Better boll opening in foliar applied K_2_SO_4_, perhaps, played decisive role for increased seed-cotton yield. For basal application and side dressing, KNO_3_ produced the highest seed-cotton yield, but the benefit cost ratio was better for foliar applied K_2_SO_4_. In crux, foliar application of K_2_SO_4_ might be opted to improve the seed cotton yield, fiber quality and net returns under the arid climate. However, soil K application through K_2_SO_4_ and/or KNO_3_ is essential to balance the K removal from soil.

## Introduction

Cotton (*Gossypium hirsutum* L.) is a cash crop grown in diverse soil types across the globe, including Pakistan. More than 100 countries of the world produce cotton over an area of 33.2 million hectare with an average annual cotton production of 18.9 million tonnes. In Pakistan, it is grown on 2.49 million hectares with an average annual production of 1.89 million tonnes [1].

Cotton productivity in Pakistan is threatened by increased pest pressure, reduced availability of certified seed and disease/pest resistant cultivars, sometime excessive rainfall at sowing time, improper cultivation method, imbalance use of fertilizers, heat stress at flowering stage and unavailability of advanced technologies [2, 3].

Optimum use of synthetic fertilizer in any crop is crucial for obtaining better crop yields and economic returns [4]. Among synthetic fertilizers, the use of K fertilizers is quite low in cotton, especially in Pakistan [5]. However, K is a vital macronutrient for plants [6], required for normal plant growth and development [7, 8]. Like ether field crops, K is essential for the growth and development of cotton crop. It is essential for many of the enzyme systems in the cotton and plays vital role in reducing the incidence and severity of the wilt disease [9]. Aneela et al. [10] reported a remarkable improvement in cotton yield and quality owning to K fertilization. It has been reported that severe K deficiency in cotton can decrease yield and reduce fiber quality by decreasing the expansion of leaf area and CO_2_ assimilation capacity [11].

The article "Efficacy of fertilizing method for different potash sources in cotton (Gossypium hirsutum L.) nutrition under arid climatic conditions" was retracted in 2022. Reasons: compromised peer review; a conflict of interest; concerns about the authorship.

The K nutrition can be improved by using appropriate K source and optimizing correct application method [7, 12]. The use of KCl is most common among various K sources owning to its relative low cost. This can also be mixed with soil or can be applied through fertigation [13]. In soil solution, KCl application releases an equal amount of K and Cl. The K entering in the soil is relatively immobile in soil solution, whereas Cl is mobile and can be easily removed through leaching [14]. However, excessive presence of Cl ion in soil solution and its later accumulation in leaves may cause toxicity. The other common K source used in crop production is K_2_SO_4_, which provides K as well as sulphur to plants [15]. Potassium nitrate (KNO_3_) is also a unique K source due to its nutritional value (as it contains 38% of K and 13% of N) [16] and higher solubility under warm conditions [17]. Its application is desirable where a relatively soluble and Cl^-^free source of K is needed [13].

The timing of K fertilizer application method depends upon fertilizer and soil type, and nature of crop [18]. The soil application of macronutrients (including K) is the most common way of improving soil fertility [19]. However, high doses of fertilizers are needed for soil application [18]. Macronutrients (such as phosphorous and K) can fix within the soil depending upon the charge of clay minerals; thus, reducing their availability to the crops. Hence alternate methods of K fertilizer application might be useful to reduce the potential losses of soil applied K fertilizers. In this scenario, foliar application of K fertilizers seems a pragmatic option to fulfil the K requirement of crops. In foliar application, the nutrient elements are easily absorbed by leaves [20]. The foliar spray of K fertilizer might be a convenient way of K supply to the plants. However, the use of excessive concentration of K can cause leaf damage [20].

The article "Efficacy of fertilizing method for different potash sources in cotton (Gossypium hirsutum L.) nutrition under arid climatic conditions" was retracted in 2022. Reasons: compromised peer review; a conflict of interest; concerns about the authorship.

Keeping in view these facts, the present study was conducted to determine the most appropriate and economical source and method of K application to improve seed-cotton yield, fiber quality and net returns of cotton sown under arid conditions.

## Material and methods

### 2.1. Site, soil and weather

This experiment was conducted at the Research Farm of Bahauddin Zakariya University, Bahadur Sub-campus, Layyah latitude 30.96^o^ N and longitude 70.93^o^ E) Pakistan during 2016. The experimental soil was sandy loam. The other physico-chemical properties of the soil are given in Table 1. The meteorological data, collected from a nearby weather station, regarding temperature and rainfall during the crop growing season is given in Fig 1.

**Fig 1:** Weather data of the experimental location during the crop season of 2016.

**Table 1:** Physio-chemical properties of the experimental site.

Soil property	Values
Soil pH	8.3
Electrical conductivity (dS m^-1^)	1.45
Available phosphorous (mg kg^-1^)	8.0
Exchangeable potassium (mg kg^-1^)	153.0
Total nitrogen (%)	0.03
Soil organic matter content (%)	0.52

### 2.2. Experimental design, experimental treatments and crop husbandry

A randomized complete block design (RCBD) with factorial arrangement (taking K sources and application methods as factors with equal importance) was followed with 03 replications and gross plot size of 3.0 m × 7.0 m. The experiment consisted of three K sources *viz*. potassium nitrate (KNO_3_), potassium sulphate (K_2_SO_4_; sulphate of potash) and potassium chloride (KCl; muriate of potash), and four K application methods *viz*. basal application (at 100 kg K_2_O ha^-1^), side dressing (at 100 kg K_2_O ha^-1^), foliar application (2%) and fertigation (at 100 kg K_2_O ha^-1^). After pre-sowing irrigation (10 cm), the experimental field was cultivated twice (with cultivator) followed by planking to prepare fine seedbed.

BT cotton cultivar Lalazar 2014 was manually sown on 75 cm spaced ridges keeping plat to plant distance of 20 cm on 20^th^ of April 2016. The ridges were made with tractor mounted ridger. The basal K application was done at the time of seedbed preparation. Foliar K application was done after 2^nd^ irrigation i.e., 8^th^ leaf emergence stage. Fertigation was done with 2^nd^ irrigation i.e., 8^th^ leaf emergence stage. Side Dressing was done after 2^nd^ irrigation. Thinning was performed at 2–4 leaf stage of the crop. Weeds were controlled manually and recommended plant protection measures were opted to keep crop free of insects and diseases. Crop was irrigated as and when required to avoid moisture stress. Management of all the experimental units was kept same except treatments and recommended agronomic practices. Crop final picking was done on November 13, 2016.

The article "Efficacy of fertilizing method for different potash sources in cotton (Gossypium hirsutum L.) nutrition under arid climatic conditions" was retracted in 2022. Reasons: compromised peer review; a conflict of interest; concerns about the authorship.

### 2.3. Data recording

The data on allometric traits were taken at 15 days interval; starting from 30 days after sowing (DAS) and terminated at crop maturity. Height of tagged plants were measured from base of the plant to tip of the main stem at fortnight intervals and averaged. Total number of opened and unopened bolls present was counted, from tagged plants and averaged. Similarly, number of sympodial and monopodial branches were counted and averaged. Weight of twenty mature bolls picked from the tagged plants was recorded and averaged to record average boll weight (g). Likewise, seed-cotton was picked up regularly from the matured bolls present in two central rows till end of October and was expressed as kg ha^−1^, as detailed in Shah et al. [3]. Seed-cotton obtained from each plot was ginned through single roller electrical gin machine and lint yield was expressed in kg ha^-1^. The ginning out turn (GOT) was calculated as;

$$GOT\;(\%)=\left(\frac{Weight\;of\;lint\;in\;sample}{Total\;weight\;of\;seed\;cotton\;in\;sample}\right)\times 100$$

The fiber quality was recorded from randomly selected clean samples of lint. For this, the lint was conditioned by placing it at 65% humidity and 18–20°C temperature in an air-conditioned chamber using humidifier. Afterwards High-Volume Instrument (HIV 900 SA) was used for determining fiber strength (μg tex^–1^), uniformity index (%), staple length (mm) and micronaire (μg/inch). Moreover, costs involved in seedbed preparation, purchasing of seed, sowing of crop, fertilizers, irrigation, crop protection measures, land rent and picking of cotton were added to estimate total production cost. Gross income was estimated according the current average market price of seed-cotton yield and cotton sticks. The benefit cost ratio (BCR) for all individual treatments was calculated by the following formula;

$$BCR=\frac{Gross\;income}{Total\;cost}$$

### 2.4. Statistical analysis

The data collected on all parameters were subjected to Fisher’s analysis of variance technique using statistical software Statistix 8.1 for the estimation of the overall significance in data, while least significant difference test at 5% probability level was used to compare differences among treatments means [21]. Pearson correlation of yield parameters with lint yield, seed-cotton yield and BCR was computed using statistical software Sigma plot 12.

## Results

The K sources and K application methods interaction significantly (p≤0.05) altered plant height, number of opened and unopened bolls per plant, boll weight, number of monopodial/sympodial branches per plant, lint and seed-cotton yield, ginning out turn, BCR, staple length, uniformity index, micronaire and fiber strength (Tables 2 and 3).

The article "Efficacy of fertilizing method for different potash sources in cotton (Gossypium hirsutum L.) nutrition under arid climatic conditions" was retracted in 2022. Reasons: compromised peer review; a conflict of interest; concerns about the authorship.

**Table 2:** Effect of sources and methods of potash application on productivity, quality and economics of cotton.

K sources/ application methods	Basal	Foliar	Fertigation	Side dressing	Basal	Foliar	Fertigation	Side dressing
	Plant height (cm)				Number of opened bolls per plant			
KCl	173 b	161 d	173 b	172 bc	31 bc	36 bc	31 bc	36 b
K_2_SO_4_	174 b	188 a	185 ab	181 ab	42 a	45 a	42 a	33 bc
KNO_3_	156 e	175 c	166 cd	173 b	31 c	35 bc	32 bc	35 bc
LSD (p ≤ 0.05)	S × M = 7.14				S× M = 5.42			
	Number of unopened bolls per plant				Average boll weight (g)			
KCl	32 a	20 b-d	23 b	18 c-f	3.25 d	3.51 ab	3.58 ab	3.38 b-d
K_2_SO_4_	17 e-f	21 b-d	19 c-e	18 c-f	3.45 b-d	3.74 a	3.38 b-d	3.40 b-d
KNO_3_	19 c-e	15 f	17 d-f	21 b-c	3.45 b-d	3.32 cd	3.51 a-c	3.29 cd
LSD (p ≤ 0.05)	S× M = 5.43				S×M = 0.25			
	Number of monopodial branches per plant				Number of **s**ympodial branches per plant			
KCl	2.7 f	3.3 a-c	2.3 f	3.3 b-d	13.0 c	13.7 bc	10.5 e	9.0 f
K_2_SO_4_	3.7 ab	4.0 a	3.0 b-e	3.4 bc	13.7 bc	15.7 a	14.5 b	11.8 d
KNO_3_	3.0 cd	2.7 d-f	2.7 ef	3.3 b-d	12.0 d	13.0 c	9.8 ef	10.3 e
LSD (p ≤ 0.05)	S×M = 0.65				S×M = 1.07			
	Lint yield (kg ha^-1^)				Seed-cotton yield (kg ha^-1^)			
KCl	639.7 f	812.2 c	684.4 e	501.01 b	1671 i	2085 d	1732 h	1165 k
K_2_SO_4_	789.1 d	904.4 ab	855.0 c	731.5 e	1915 f	2343 a	2208 c	1900 fg
KNO_3_	762.0 d	925.5 a	597.0 b	781.9 d	2016 e	2334 a	1584 j	2326 ab
LSD (p ≤ 0.05)	S×M = 35.8				S×M = 17.2			
	Ginning out turn (%)				Benefit cost ratio			
KCl	38.1 cd	39.1 ab	39.4 ab	39.4 ab	1.11 c	1.10 c	1.14 c	1.00 e
K_2_SO_4_	41.1 a	38.6 cd	38.7 bc	38.5 cd	1.12 c	1.30 a	1.08 cd	1.05 d
KNO_3_	36.2 d	39.7 ab	37.6 cd	33.7 e	1.00 e	1.24 b	1.20 b	1.03 d
LSD (p ≤ 0.05)	S × M = 2.5				S × M = 0.05			

Means of interactions not sharing a same case letter for a parameter differ significantly at p ≤ 0.05

K_2_SO_4_ = sulphate of potash, KCl = muriate of potash; KNO_3_ = potassium nitrate

**Table 3:** Effect of sources and methods of potash application on fiber quality of cotton.

K sources/ application methods	Basal	Foliar	Fertigation	Side dressing	Basal	Foliar	Fertigation	Side dressing
	Staple length (cm)				Uniformity index (%)			
KCl	28.1 f	29.5 c	28.7 e	28.6 e	82.4 d	84.3 c	84.1 c	82.5 d
K_2_SO_4_	28.9 de	31.5 a	31.4 a	30.4 b	84.7 bc	86.9 a	86.8 a	86.7 a
KNO_3_	28.8 e	29.4 c	29.3 cd	28.6 e	84.5 c	84.2 c	85.2 b	82.9 d
LSD (p ≤ 0.05)	S × M = 0.38				S× M = 0.66			
	Micronaire (μg/inch)				Fiber strength (g/tex)			
KCl	3.7 de	4.0 bc	3.8 c-e	3.5 f	26.0 g	26.4f g	29.6 b	29.6 b
K_2_SO_4_	3.7 d-f	4.4 a	3.9 b-d	4.0 bc	29.3 bc	30.8 a	29.4 b	28.1 de
KNO_3_	4.1 b	3.6 ef	3.9 b-d	3.8 c-e	27.2 ef	28.4 cd	27.8 de	26.5 fg
LSD (p ≤ 0.05)	S× M = 0.22				S×M = 0.98			

Means of interactions not sharing a same case letter for a parameter differ significantly at p ≤ 0.05

K_2_SO_4_ = sulphate of potash, KCl = muriate of potash; KNO_3_ = potassium nitrate

The highest plant height was recorded with foliar application of K_2_SO_4_ and that was statistically similar with fertigation and side dressing of K_2_SO_4_ (Table 2). The highest number of opened boll per plant was also recorded with foliar application of K_2_SO_4_, which was statistically similar with the basal application and side dressing of K_2_SO_4_ (Table 2). The highest number of unopened bolls was recorded with the basal application of KCl, whereas minimum was noted with foliar application of KNO_3_ (Table 2). The highest boll weight was recorded with foliar application of K_2_SO_4_ and that was statistically similar with fertigation of KCl (Table 2). The highest number of monopodial and sympodial branches per plant was recorded with the foliar application of K_2_SO_4_ and that was statistically similar with basal application of K_2_SO_4_ for number of monopodial branches per plant (Table 2). Lint and seed-cotton yield, and BCR was also highest with foliar applied K_2_SO_4._ However, ginning our turn was the highest with basal application of K_2_SO_4_ (Table 2). The staple length, uniformity index, micronaire and fiber strength was the highest with foliar application of K_2_SO_4_; and that was statistically similar with fertigation of K_2_SO_4_ for staple length with fertigation and side dressing of K_2_SO_4_ for uniformity index (Table 2). We observed a strong positive correlation of opened bolls per plant, boll weight per plant, monopodial and sympodial branches with lint yield, seed-cotton yield and BCR (Table 4).

The article "Efficacy of fertilizing method for different potash sources in cotton (Gossypium hirsutum L.) nutrition under arid climatic conditions" was retracted in 2022. Reasons: compromised peer review; a conflict of interest; concerns about the authorship.

**Table 4:** Co-relation coefficients of growth and yield parameters with lint yield, seed cotton yield and benefit cost ratio.

Crop Variables	Lint yield	Seed cotton yield	Benefit-cost ratio
Number of bolls per plant	0.81*	0.81*	0.89**
Average boll weight	0.86*	0.85*	0.83*
Monopodial branches	0.90**	0.88*	0.87*
Sympodial branches	0.91**	0.97**	0.93**

* = significant at p ≤ 0.05

** = significant at p ≤ 0.05

## Discussion

This study indicated that application of K through various sources coupled with different application methods significantly affected all measured allometric, yield and quality related traits (Tables 2 and 3).

Improvement in seed cotton yield and quality due to K application might be attributed to K involvement in several metabolic processes of crop plants. For example, use of K in cotton decreases the severity and incidence of wilt diseases, improves water use efficiency and fiber quality (in terms of micronaire, fiber length/strength) by maintaining surplus water pressure within the boll [22]. On the other hand, K shortage in cotton may decrease fiber quality by exposing the plants to water stress and diseases [22]. Moreover, the improvement in cotton performance due to K application might be attributed to the increased photosynthetic rate owing to role of K in CO_2_ fixation and cell turgor control [23]. The K application in cotton is also believed to extend N absorption, which causes vigorous vegetative growth [19] and ultimately increases yield. The use of K fertilizers in cotton enhanced metabolic activity and improved staple length, tensile strength, fiber micronaire, and decreased the amount of damaged fiber [24]. Several other studies have reported an improvement in seed-cotton yield and fiber quality due to K application in cotton [4, 10, 25, 26].

Among various K sources used, K_2_SO_4_ was comparatively better option to improve the morphological/yield parameters, seed-cotton yield and fiber quality. Indeed, K_2_SO_4_ contains sulfur besides K, which enhances protein synthesis, enzyme functioning, and cell elongation [26], ultimately improves crop yield as observed in this study. Moreover, the use of K_2_SO_4_ has been found to improve vegetative growth [27], lint yield, and quality of cotton [28, 29, 30] through reduction in the number of unopened bolls and an improvement in the number of opened bolls per plant as compared with other K sources. The highest seed-cotton yield due to foliar applied K_2_SO_4_ in this study might be attributed to the improvement in boll weight, number of opened bolls per plant and more number of monopodial and sympodial branches (Tables 2 and 4).

The use of KCl was not a better option to improve cotton yield and fiber quality under arid conditions of Layyah. Indeed, KCl contains chlorides which are already present in enough quantities in the soils of arid regions [31]. Thus, excessive addition of Cl from KCl may enhance the Cl^-^ level in soil, which negatively impacts cotton yield and quality.

Foliar application of K_2_SO_4_ was found beneficial for improvement in seed-cotton yield and fiber quality. Indeed, foliar application of macronutrients ensures direct absorption; thus, minimizing leaching losses and fixation as happens in soil application. Several other studies have reported improvement in cotton yield due to foliar K application [29, 32, 33, 34].

The highest net benefits were recorded with the foliar application of K. Indeed, very small amount of a fertilizer is required for foliar application which decreases input cost incurred on fertilizer purchase. Moreover, higher seed-cotton yield due to foliar application enhanced the output in terms of monetary turns, which enhanced the probability of cotton with foliar application. Some other studies have reported that foliar application of K enhanced the net benefits [35]. However, high rates of K fertilization may cause leaf burn which should be kept in mind when opting foliar application method under field conditions. Importantly, foliar application will not be the best option always, because it will not fulfil the nutritional requirements under K-deficient conditions. In this study soil had >150 mg K kg^-1^ soil which is considered as sufficient K content for most of the crops; however, foliar K application contributed some extra benefits due to timely and direct K application when required by plants in very large amounts and soil supply of K may not be sufficient [29, 30].

The article "Efficacy of fertilizing method for different potash sources in cotton (Gossypium hirsutum L.) nutrition under arid climatic conditions" was retracted in 2022. Reasons: compromised peer review; a conflict of interest; concerns about the authorship.

In conclusion, foliar application of K_2_SO_4_ seemed a viable option to harvest higher seed-cotton yield along with better quality fiber, and higher returns of cotton sown under arid conditions.
